# Effects of head positions on awake fiberoptic bronchoscope oral intubation: a randomized controlled trial

**DOI:** 10.1186/s12871-021-01397-4

**Published:** 2021-06-23

**Authors:** Zhuo Liu, Li Zhao, Zhongfeng Ma, Meiqi Liu, Xiaohang Qi, Qianqian Jia, Shujuan Liang, Xiaochun Yang

**Affiliations:** 1 Department of Anesthesiology, the First hospital of Qinhuangdao, N.O. 258, Wenhua Road, Qinhuangdao, Hebei China; 2 Department of thoracic surgery, the First hospital of Qinhuangdao, N.O. 258, Wenhua Road, Qinhuangdao, Hebei China; 3 Department of general surgery, the First hospital of Qinhuangdao, N.O. 258, Wenhua Road, Qinhuangdao, Hebei China

**Keywords:** Awake orotracheal intubation, Fiberoptic-bronchoscope, Head positions

## Abstract

**Background:**

There are many factors affecting the success rate of awake orotracheal intubation via fiberoptic bronchoscope. We performed this study was to investigate the effects of head positions on awake Fiberoptic bronchoscope oral intubation.

**Methods:**

Seventy-five adult patients, received general anaesthesia were included in this study. After written informed consent, these patients were undergoing awake orotracheal intubation via fiberoptic-bronchoscope and according to the head position, the patients were randomized allocated to neutral position group (NP group), sniffing position group (SP group) or extension position group (EP group). After sedation the patients were intubated by an experienced anesthesiologist. The time to view the vocal cords, the percentage of glottic opening scores (POGO), the time to insert the tracheal tube into trachea and the visual analog scale (VAS) scores for ease experienced of passing the tracheal tube through glottis, the hemodynamic changes and the adverse events after surgery were recorded.

**Results:**

The time to view the vocal cords was significantly shorter and the POGO scores was significantly higher in the EP group compared with the other two groups (*P* < 0.05); The SpO_2_ in the EP group was higher than NP group at before intubation and higher than SP group and NP group at immediate after intubation (*P* < 0.05); The time to insert the tracheal tube into trachea, the VAS scores for passing the tracheal tube through glottis, the coughing scores had no significant differences among groups (*P* > 0.05). There were also no significant differences regard to the incidence of postoperative complications, mean arterial pressure and heart rate among the groups (*P* > 0.05).

**Conclusions:**

The head at extension position had a best view of glottic opening than neutral position or sniffing position during awake Fiberoptic bronchoscope oral intubation, so extension position was recommended as the starting head position for awake Fiberoptic bronchoscope oral intubation.

**Trial registration:**

Clinical Trials.gov. no. NCT02792855. Registered at https://register.clinicaltrials.gov on 23 september 2017.

## Background

The incidence of difficult airway is ranging from 0.3 to 13% [1] and nearly 30% of all anaesthesia-related deaths are attribute to difficult airway [2]. Awake tracheal intubation via Fiberoptic bronchoscope (FOB) is regarded as the golden standard for the management of difficult airway [3–6]. However, in sedated patients, the base of tongue, soft palate and epiglottis move backward and obstruct the advancement of FOB [7, 8]. Recently, several studies have examined the effects of different methods such as jaw thrust, lingual traction or head tilt on FOB intubation [9–15]. However, there have been no study to determine which head position (neutral position, sniffing position or extension position) is the most suitable for Awake Fiberoptic bronchoscope oral intubation (AFOI). Thus, the objective of this study was to investigate the effects of three head positions during AFOI.

## Methods

This trial was approved by the institutional review board of the first hospital of Qinhuangdao and all patients provided written informed consent.

Seventy-five adult patients, ASA class I-II, modified Mallampati classification ≥3, requiring general anaesthesia and undergoing awake orotracheal intubation were included in this study. Exclusion criteria were as follows: age > 70 or < 18 years, with cervical spine disease, loose or missing incisors, preoperative hoarseness, bronchial asthma, a history of airway hyperreactivity, hypertension and abnormalities of heart, brain, liver, lung, kidney and coagulation functions.

All these patients were screened by the same senior anaesthesiologist preoperatively and according to the head position, the patients were randomized allocated to neutral position group (NP group: with the occiput close to the operating table, Fig. 1A), sniffing position group (SP group: with a 7-cm pillow underneath the occiput, Fig. 1B) or extension position group (EP group: with a 7-cm pillow underneath the shoulder and the occiput close to the operating table, Fig. 1C). Randomization (1:1:1) was based on the codes generated by Excel software, which were kept in sequentially numbered opaque envelopes until the began of study. (Fig. 2).

**Fig. 1:** The position of intubation was demonstrated by a volunteer: **A**, ‘neutral’ position with the occiput close to the operating table; **B**, ‘sniffing’ position with a 7-cm pillow underneath the occiput; **C**, ‘extension’ position with a 7-cm pillow underneath the shoulder and the occiput close to the operating table

**Fig. 2:** Flow diagram

All the patients without premedication and received standard monitoring systems, including electrocardiogram (ECG), heart rate (HR), non-invasive arterial blood pressure (NIBP) and peripheral oxygen saturation (SpO_2_) in the operating room. The patients were intravenously injected with midazolam 0.03 mg·kg^− 1^. After mild sedation, a intratracheal injection was performed at the cricothyroid membrane with a fine needle and administered with 2% lidocaine (3-4 ml), then the patients were suggested to open the mouth as wide as possible and then the oral cavity and hypopharynx mucosa were sprayed with 2% lidocaine (1-2 ml). After intratracheal anaesthesia, dexmedetomidine was administered at a loading dose of 1 μg·kg^− 1^ (the infusion was completed in 10 min) then remifentanil was given at a loading dose of 0.5 μg·kg^− 1^, followed by a continuous infusion at a speed of 0.1–0.15 μg·kg^− 1^·min^− 1^. During this process the patients received continuous oxygen by mask at a rate of 5 L/min.

Before intubation, a FOB (external diameter 5.2 mm, MDHAO Medical Technology Co, Ltd., Zhuhai, China) was loaded with a silicone flexible tracheal tube (Tuoren Medical Technology Co, Henan, China: inner diameter 6.5 mm for female and 7.0 mm for male) and lubricated with dyclonine hydrochloride mucilage. After sedation to Ramsay Sedation Score (RSS) of 3 or 4 [16], the intubation was performed and the steps were as follows: First, a bite block was placed between the teeth of patients then the operator holded the control section of the FOB with his right hand and inserted the anterior of FOB into the mouth with his left thumb and left index finger, simultaneously gripped the chin upward with the remaining fingers. At this point, the bite block as a fulcrum to lift the mandible upward to open the space of pharynx and laryngeal cavity as far as possible (Fig. 1A, B, C) then advanced the FOB downward along the oropharyngeal curve with his left thumb and left index finger until viewing the epiglottis and glottis. After the anterior of FOB passed through the vocal cords, the FOB was inserted into the trachea and then the tracheal tube was slipped gently into the trachea over the FOB. AFOI was suspended when SpO_2_ < 90% and oxygen was supplied by mask. If AFOI has not been successful more than three times, we would stop the intubation and alternate to a laryngeal mask or a laryngeal tube [17] and wake the patient as quickly as possible.

The primary outcome parameters of the study were the time to view the vocal cords (TVVC) and the percentage of glottic opening scores (POGO). TVVC was defined as the time from inserting the FOB between the teeth until the operator view the the entire vocal cords; POGO scores (score range:0–100: 0 = none, 100 = full) [18, 19] was defined as the operator’s first vision of glottic opening during the FOB just passed the tongue base. The time to advance the tracheal tube into trachea over FOB (TATT) defined as the time from viewing the entire vocal cords to insert the tracheal tube into trachea successfully, the coughing scores (score range: 0 = none, 1 = slight, 2 = moderate, 3 = severe) [20] when inserted the FOB into trachea and inserted the tracheal tube into trachea via FOB, the VAS scores (score range:0–100, 0 = very difficult, 100 = very easy) of the ease experience for inserting the tracheal tube into trachea indicated by the operator immediately after the intubation, the hemodynamic changes of patients during intubation and postoperative complications such as hoarseness and throat pain were also recorded. TVVC, TATT and POGO scores were assessed by an independent observer.

In our study, the sample size was determined according to a pilot study, with significance set at 0.05 and power set at 80%, the sample size required to detect the differences of the POGO scores was 20 patients each group. Taking into account that the potential risk of patients excluded from the study for unforeseen reasons we recruited 25 patients each group.

Analyses were performed using SPSS 21.0 statistical software. Continuous variables were presented as mean ± standard deviation (SD) and the differences among the groups were compared with ANOVA test. The differences of proportions were analyzed using Kruskal-Wallis test. The differences of the incidence were analyzed with Fisher’s exact test. *P* value less than 0.05 was considered as statistically significant.

## Results

There were no significant differences in the demographic characteristics, thyromental distance, mallampati class, mouth opening and degree of neck extension among groups (Table 1).

**Table 1:** Demographic characteristics of patients

Characteristics of patients	SP (*n* = 25)	NP (*n* = 25)	EP (*n* = 25)	*P*-value
Age (years)	50.8 ± 13.2	51.0 ± 11.1	53.9 ± 10.3	0.58
Gender (M/F, n)	11/ 14	14/11	13/12	0.68
ASA (I/II, n)	15/10	12/13	14/11	0.32
Weight (kg)	68.9 ± 16.2	70.7 ± 9.9	70.5 ± 11.9	0.87
Height (cm)	165.1 ± 9.0	166.9 ± 6.8	167.4 ± 7.8	0.58
BMI (kg/m^2^)	25.1 ± 4.2	25.4 ± 3.3	25.1 ± 3.4	0.95
Thyromental distance (cm)	5.1 ± 0.6	5.5 ± 0.5	5.2 ± 0.9	0.26
Mouth opening (cm)	4.5 ± 0.9	4.4 ± 1.5	4.2 ± 1.1	0.73
Mallampati class (3 /4, n)	12/13	9/16	11/14	0.68
Degree of neck extension				0.49
> 90°(n)	21	24	23	
≤ 90°(n)	4	1	2	

*ASA* American Society of Anesthesiologists, *BMI* Body mass index; Statistical analysis indicated no significant differences in the parameters among groups (*P* > 0.05)

The time to view the vocal cords was significantly shorter and the POGO scores was significantly higher in the EP group compared with the other two groups (*P* < 0.05); The time to tracheal intubation, the VAS scores for passing the tracheal tube through glottis, the incidence of postoperative complications, the coughing scores when inserted FOB into the trachea and inserted the tracheal tube into the trachea over FOB had no significant differences among groups (*P* > 0.05) (Table 2).

**Table 2:** Comparison of the time to view the vocal cords, time to advance tracheal tube into trachea, percentage of glottic opening scores, the VAS scores for ease of passing the tracheal tube through the glottis, the coughing scores and the adverse events after tracheal intubation

Factor	SP (*n* = 25)	NP (*n* = 25)	EP (*n* = 25)	*P*-value
Time to view the vocal cords (TVVC) (s)	20.1 ± 9.9	22.5 ± 10.5	14.2 ± 4.9^*#^	< 0.01
Time to advance tracheal tube into trachea (TATT) (s)	17.4 ± 5.8	19.8 ± 9.6	17.5 ± 8.1	0.51
Percentage of glottic opening scores (POGO) (%)	78.5 ± 20.5	75.2 ± 19.6	88.9 ± 11.5^*#^	0.02
VAS scores for tracheal tube passing glottis	87.4 ± 13.7	79.3 ± 23.5	82.4 ± 19.4	0.33
Coughing scores of inserting FOB (0/ 1 /2/ 3, n)	23/2/0/0	22/2/1/0	24/1/0/0	0.94
Coughing scores of inserting tracheal tube (0/ 1 /2/ 3, n)	12/5/7/1	11/7/4/3	14/7/2/2	0.98
Throat pain(n)	6	6	8	0.76
Hoarseness (n)	1	2	1	0.77

*VAS* Visual analog scale (score range, 0–100, score 0 = very difficult, 100 = very easy); Coughing score (score range, 0 = none, 1 = slight, 2 = moderate, 3 = severe) ^*^P < 0.05 compared with SP group, ^#^*P* < 0.05 compared with NP group

The SpO_2_ in the EP group was higher than NP group at before intubation and higher than SP group and NP group at immediate after intubation (*P* < 0.05), while at other time points the SpO_2_ had no significant difference among groups (*P* > 0.05). There were no significant differences among the groups with regard to mean arterial pressure and heart rate during intubation (*P* > 0.05) (Table 3).

**Table 3:** Hemodynamic alterations of patients during intubation

Factor	SP (*n* = 25)	NP (*n* = 25)	EP (*n* = 25)	*P*-value
MAP (mmHg)				
T0	96.3 ± 10.2	101.2 ± 9.5	100.0 ± 11.1	0.22
T1	91.1 ± 13.5	92.3 ± 12.2	97.4 ± 11.2	0.18
T2	97.8 ± 14.8	100.0 ± 14.6	105.8 ± 13.4	0.13
T3	91.3 ± 14.8	95.7 ± 13.4	98.5 ± 13.5	0.18
T4	87.5 ± 13.5	90.2 ± 14.3	94.4 ± 11.9	0.21
HR (bpm)				
T0	74.1 ± 13.4	72.8 ± 13.4	75.7 ± 8.7	0.71
T1	67.3 ± 12.8	64.8 ± 10.9	66.3 ± 10.8	0.74
T2	71.2 ± 15.1	64.6 ± 10.6	64.4 ± 11.6	0.11
T3	65.6 ± 11.3	61.7 ± 10.0	62.4 ± 11.7	0.40
T4	65.4 ± 12.4	60.9 ± 8.4	62.2 ± 11.0	0.33
SpO_2_ (%)		–		
T0	97.5 ± 1.6	98.1 ± 1.8	98.5 ± 1.5	0.10
T1	97.7 ± 2.4	96.4 ± 3.5	98.8 ± 2.0^#^	0.01
T2	96.4 ± 5.1	97.6 ± 2.2	99.1 ± 1.4^*#^	0.02
T3	98.8 ± 2.1	98.8 ± 2.4	99.6 ± 0.6	0.20
T4	99.5 ± 0.7	99.3 ± 1.4	99.2 ± 1.5	0.73

*MAP* Mean arterial pressure, *HR* Heart rate, *SpO*_*2*_ pulse oxygen saturation, *T0* Before anesthesia, *T1* Before intubation, *T2* Immediate after intubation, *T3* 1min after intubation, *T4* 3min after intubation. ^*^P < 0.05 compared with SP group, ^*#*^*P* < 0.05 compared with NP group

## Discussion

In this study, we compared the effects of three head positions (neutral position, sniffing position and extension position) during AFOI. The results showed us that the POGO scores were significantly higher and the time for viewing the whole vocal cords was significantly shorter in the EP group compared with the other two groups. The results slao showed us that the SpO_2_ in the EP group was higher than NP group at before intubation and higher than the SP group and NP group at immediate after intubation. The reasons may be that although the anterior of FOB can cross the angle among the three axes (oral axes, pharyngeal axes and laryngeal axes) [21, 22], FOB can not provide enough support to the laryngeal tissue, resulting in the base of tongue, soft palate and epiglottis were closer to the posterior pharyngeal wall [23], lead to the operator unable to find the glottis easily in sedated patients using FOB. In present study, all the patients in the EP group with heads at extension positions by placing a 7-cm firm pillow under the shoulders, so this positions tightened the muscles and tissues in the front of neck then moved the oropharyngeal structures anteriorly and emptied the oropharyngeal airspace. So the extension position was better than the other two positions to keep the airway open in sedated patients and maked it easier for the FOB to pass through the base of the tongue and easier to view the whole glottis.

Several studies found that the manoeuvre of jaw-thrust [10–15], the combining used of jaw thrust and lingual traction [11], the combining used of FOB and laryngoscopy technique [12] can elevated the epiglottis and tongue base away from the wall of posterior pharyngeal, provided more space in the pharyngeal cavity and laryngeal cavity, which facilitated the operator to view the vocal cords and increased the success rate of oral intubation by FOB [24]. The problem with these methods was that one or two trained assistants were required. In this study, the operator made the bite block as a fulcrum and lifted the mandible upward more easily than other two positions during intubation, which may achieve similar effects as jaw thrust that enabling the FOB easily to pass through the base of the tongue. Most important one was that the whole process of intubation without the assistance by others.

Successful inserting a FOB into the trachea does not guarantee a successful AFOI, because the anterior of the tracheal tube may impinge on the laryngeal structures when advance the tracheal tube into trachea over the FOB [25, 26], which may lead to serious injury of laryngeal [27] or be catastrophic in some cases [15]. This difficulty can be reduced by reducing the gap between the tracheal tube and FOB [28]. In this study, the outside diameter of FOB was 5.2 mm and the inner diameter of tracheal tube was 6.5 mm for female and 7.0 mm for male, so the gap between the tracheal tube and FOB was very small, furthermore we used silicone flexible tracheal tube and the inside and outside of the tracheal tube was lubricated with dyclonine hydrochloride mucilage, so the advancement of a tracheal tube over the FOB very smoothly.

In our study, all the patients were unable to recall the procedure of intubation and the hemodynamic changes, coughing scores had no statistical differences among groups, the reasons may be that topical anaesthesia of the trachea and the combined use of dexmedetomidine and remifentanil not only preserved the patients’ spontaneous breathing but also achieve adequate sedation depth during intubation to reduced the incidence of adverse complications and improved the comfort of patients [29].

There were also some limitations in our study. First, this method is not suitable to patients with disorder of cervical spine; Second, this method is not suitable to patients with incisors loose or missing for the operator unable to lifted the mandible upward using the bite block as a fulcrum; Third, this method may not be applicable to the patient with oversize-chin or the operator with little experience in the management of FOB; Fourth, subjective scales were used to assess the outcomes; Fifth, it was not possible to blind investigator to the technique, consequently we cannot rule out the possibility of biases by investigator in this study.

## Conclusion

Extension position had a better view of glottic opening than neutral position or sniffing position during AFOI, so extension position may be recommended as the initial head position for AFOI.

## Data Availability

The datasets are available from the corresponding author on request.

## Abbreviations

POGO: Percentage of glottic opening scores
VAS: Visual analog scale scores
ASA: America society of anesthesiology
FOB: Fiberoptic bronchoscope
AFOI: Awake Fiberoptic bronchoscope oral intubation
TVVC: Time to view the vocal cords
TATT: Time to advance the tracheal tube into trachea over FOB
SPSS: Statistical package for social sciences
